# Expression and Relationship of Netrin-1, DCC, UNC5B, and VEGF in Villous Tissues of Patients with Delayed Abortion

**DOI:** 10.1155/2022/6283372

**Published:** 2022-08-30

**Authors:** Fen Dong, Yan Cao, Zhonghui Huang, Sha Li

**Affiliations:** ^1^Huai'an Maternal and Child Health Care Center, Huai'an 223001, China; ^2^Department of Breast Thyroid and Vascular Surgery, The Affiliated Huai'an Hospital of Xuzhou Medical University and the Second People's Hospital of Huai'an, Huai'an 223001, China; ^3^Department of Science and Education, LianshuiPeople's Hospital, Huai'an 223001, China

## Abstract

In order to investigate the correlation between neuroaxon-guiding factor (Netrin-1), deleted in colorectal cancer (DCC), uncoordinated 5B (UNC5B), and vascular endothelial growth factor (VEGF) expression machine in villus tissues of delayed abortion in colorectal cancer, a total of 120 pregnant women are selected from February 2019 to August 2021. The two groups of subjects improve the relevant examinations before surgery and the underwent negative pressure induces abortion hysterectomy guided by abdominal ultrasound under intravenous anesthesia. The mRNA and protein expressions of netrin-1, DCC, UNC5B, and VEGF in the villi of the two groups are detected by real-time fluorescence quantitative polymerase chain reaction (RT-PCR) and immunohistochemistry (IHC), and the correlation of the four indicators is analyzed by Pearson's test.

## 1. Introduction

Missed abortion (MA) occurs 20 weeks before gestation, when the fetus or embryo died but remained in the uterine cavity without natural discharge [1]. It can lead to decreased fertility and threaten the life safety of pregnant women [2]. In recent years, diseases caused by uterine and placental vascular circulation disorders have been attached great importance in the field of perinatal medicine. Some scholars have studied the influencing factors of fetal growth restriction (FGR) and uterine and placental circulation disorders in preeclampsia, but there are few studies on early pregnancy and delayed abortion. Some studies have confirmed that vascular endothelial growth factor (VEGF) and other proangiogenic factors are related to placental angiogenesis [3, 4]. In addition, netrin-1 and its receptor deleted in colorectal cancer and uncoordinated 5B (unc5b), both of which are novel angiogenesis regulators [5]. UNC5B was gradually discovered.

In recent years, the research on the pathogenesis of delayed abortion has made great progress in the aspects of genetics, immunology, infection, and environment. Good formation of placental vascular network plays an extremely important role in fetal intrauterine development [6]. If the insufficient placental vascular dysplasia, perfusion, and placental microcirculation dysfunction can lead to placental insufficiency, placenta implantation dysfunction, maternal oxygen, nutrients, and immune factors cannot enter the fetal body through vascular network [7]. In recent years, the role of neuroaxon-guiding factor (Netrin-1) and its receptors deleted in colorectal Cancer (DCC) and UNC5B in placental circulation have attracted more attention. The expression of various factors maintaining the placenta of pregnancy is coordinated and affects each other, and the imbalance can lead to insufficient placenta angiogenesis and increase the probability of delayed abortion.

This study analyzes the expressions of netrin-1 and its receptors DCC, UNC5B, and VEGF in MA villous tissues, and the possible roles of each factor in the occurrence of delayed abortion. The expressions of netrin-1, DCC, and VEGF are low in villous tissues of patients with aborted abortion, while the expressions of UNC5B are high. The abnormal expressions of the four indicators may be related to the formation disorder of villous vessels in aborted abortion, and the changes of netrin-1, DCC, UNC5B, and VEGF indicators are closely related.

The rest of this paper is organized as follows.  Section 2 discusses related work.  Section 3 contains descriptions of data and methods.  Section 4 shows the experimental results, and Section 5 discusses and concludes this paper.

## 2. Related Work

Villus tissue detection in this study showed that compared with the control group, the protein and mRNA expressions of netrin-1, DCC, and VEGF in the aborted abortion group were decreased, while the protein and mRNA expressions of UNC5B were increased. Netrins are highly expressed in the nervous system of almost all species. Studies have shown that netrins have great similarity with the extracellular matrix protein laminin [8]. Netrin-1, a member of the Netrins family, has a typical dual orientation, which can be activated when the axonal growth cones of nerve cells reflect different receptors. The structure of netrin-1 receptors can be classified into two types: the first is DCC and the second is UNC5 homologue (UNC5H) [9].

Some studies have speculated that there may be many same signaling factors involved in nerve distribution and vascularization of vascular bodies [10]. There are no nerves in the placenta, but during the development of placental villi, a neuro-like structure will be formed. Some studies have confirmed that netrin-1 axis plays a certain role in the growth and development of cells. In addition, netrin-1 is found in the third-level villous vascular endothelial cells of placenta, which plays a certain role in cell growth [11]. Some scholars have studied the influencing factor netrin-1 and its receptor DCC and UNC5B in FGR and hysteroplacental circulation disorders of preeclampsia. The results showed that netrin-1 and its receptor DCC were in low expression and UNC5B was in high expression in the placental tissues of the abovementioned lesions. Local netrin-1 in the placenta is more likely to affect the growth of the placental vascular network, resulting in too small placental blood vessel area and failure of placental blood supply to maintain fetal growth, leading to diseases. Low expression indicates that normal placental circulation is prevented and may result in an abortive abortion. The high expression of UNC5B in delayed abortion indicates that UNC5B may be a negative regulator and may inhibit the growth and development of placental blood vessels, which may cause delayed abortion. VEGF, a glycoprotein, has a significant effect on vascular endothelial cells and is the target of hypoxia-inducible factor (HIF-L*α*). VEGF regulates angiogenesis by promoting endothelial cell function in the process of angiogenesis. VEGF family is known to be an important factor in regulating placental angiogenesis [12].

The combined transplantation of netrin-1 and mesenchymal stem cells (MSCs) in the rat model of hind limb ischemia shows that netrin-1 could significantly improve the cell migration, lumen formation ability, and vascular density of MSCs in ischemic area. Therefore, the effect of stem cell therapy on ischemic diseases can be improved, and the reperfusion and injury repair of ischemic sites can be promoted. At this point, the plasma VEGF level is also increased correspondingly [13]. In conclusion, netrin-1 can not only directly induce angiogenesis by regulating the biological function of endothelial cells but also promote the secretion of VEGF under the stimulation of pathological environment such as ischemia and hypoxia, and synergistically accelerate angiogenesis. Pearson correlation analysis showed that there is no correlation between netrin-1, DCC, UNC5B, and VEGF mRNAs in the control group [14]. In the study group, netrin-1 is negatively correlated with UNC5B and directly proportional to DCC. Netrin-1 is directly proportional to VEGF. DCC is negatively correlated with UNC5B. DCC is positively correlated with VEGF, and UNC5B is inversely proportional to VEGF. According to the abovementioned correlation analysis, netrin-1, DCC, and VEGF played a coordinating role in placental vasogenesis, while UNC5B antagonizes the abovementioned factors [15]. It is speculated that the expression of various factors regulating placental formation of normal pregnancy is in coordination with each other. If the state cannot be kept in balance, it will lead to be insufficient placental angiogenesis and increase the probability of delayed abortion. If the negative regulation of netrin-1 receptor pathway is dominant, angiogenesis may be blocked and delayed abortion may occur. Whether such changes in netrin-1 family expression in embryonic stopped, villi are the cause or result of abnormal angiogenesis of embryonic stopped. Villi remains to be further studied.

## 3. Data and Methods

### 3.1. General Information

From February 2020 to August 2020, 30 patients diagnosed with delayed abortion treated in the outpatient department of family Planning of our hospital are included in the study group. The inclusion criteria are as follows: (1) age between 20 and 34; (2) 8 to 12 weeks of gestation; (3) regular menstruation and accurate last menstruation time; (4) MA confirmed by color ultrasound examination [5]; and (5) no experience of taking hormone drugs during pregnancy and no experience of mifepristone and misoprostol medical abortion before surgery. The exclusion criteria are as follows: (1) irregular menstrual cycle; (2) abnormal reproductive tract structure; (3) genital tract infections such as *Chlamydia trachomatis* and *Ureaplasma urealyticum*; (4) patients with uterine fibroids and adenomyoma; (5) pregnancy with IUD; (6) elderly pregnant women, age ≥ 35 years old, and thyroid disease. During the same period, 60 normal early pregnant women with unwanted pregnancy waiting for pregnancy termination operation were used as the control group. Inclusion criteria are as follows: (1) gestational age between 8 and 12 weeks, regular normal menstruation, and accurate last menstruation; (2) serum HCG was positive; (3) color ultrasound examination showed pregnancy bud and cardiac tube pulsation, embryo survival, and gestational sac size consistent with the time of menopause; and (4) no previous adverse pregnancy and childbirth experience. All pregnant women signed informed consent and the study is approved by the ethics Committee of the hospital. There is no difference in general data between the two groups (*P* > 0.05). Baseline data comparison is shown in Table 1.

### 3.2. Methods

#### 3.2.1. Specimen Collection and Processing Methods

The two groups of subjects improve in the relevant examinations before surgery, and the underwent negative pressure induces abortion hysterectomy guided by abdominal ultrasound under intravenous anesthesia. The components are quickly separated from the sucked villous tissue, and one of them is frozen at −80°C for PCR detection, while the other was fixed at 4% formalin for IHC detection.

#### 3.2.2. Expressions of Netrin-L mRNA, DCC/UNC5B mRNA, and VEGF mRNA

Total mRNA is extracted from the villus tissue according to the instructions of the total RNA extraction kit and is reversely transcribed into cDNA for PCR amplification. PCR reaction conditions: pre-denaturation at 95°C for 3 min, denaturation at 95°C for 10 s, annealing at 58°C for 30 s, extension at 72°C for 30 s, and 40 cycles. PCR products are subjected to 1% agar-gel electrophoresis. GAPDH is used as a standardized internal reference. The expression of netrin-1, DCC/UNC5B, and VEGF is quantified by 2^−△△Ct^ compared with *Ct*. Gene primer sequences are shown in Table 2.

#### 3.2.3. Expressions of Netrin-1, DCC, UNC5B, and VEGF in Villous Tissues Detected by IHC

The villous tissues fixed with 4% formaldehyde fixative are prepared, sectioned, dehydrated, waxed, and embedded. Endogenous peroxidase is blocked by hydrogen peroxide and sealed by serum. Netrin-1 (1 : 100), DCC (1 : 200), UNC5B (1 : 200), and VEGF (1 : 200). The primary antibody is placed in a wet box at 4°C and incubated for 15 h. The enzyme-conjugate secondary antibody is added and incubated at 37°C for 20 min. A color developing agent is added to redyeing, dehydration, and tablet sealing. In the negative control, the drops are changed from primary antibody to PBS, and microscopic examination was taken. Five fields are randomly selected under the microscope. Image dyeing intensity is analyzed by IM-AgePro Plus 6.0 software(Media Cybernetics, USA). IHC staining intensity is expressed as integrated option density (IOD). The larger OD value, the stronger the positive reaction.

#### 3.2.4. Statistical Methods

SPSS19.0 statistical software is used for statistical analysis. *t* test was used for measurement data and all measurement data are expressed as mean ± standard deviation (‾*x* ± *s*). An OVA is used, and the rate of count data (%) is expressed. The comparison of the rates between the two groups is performed by *χ*^2^ test, *P* < 0.05 is considered statistically significant. We use Pearson's test to determine data correlation.

## 4. Experimental Result

### 4.1. Differences in PCR Detection Results of the Four Indicators

Compared with the control group, only UNC5B mRNA is upregulated in the study group and the other three indicators are significantly decreased, with statistically significant differences (*P* < 0.05). The PCR results of the four indexes are shown in Table 3.

### 4.2. Correlation between the mRNA Expression of Netrin-1, DCC, UNC5B, and VEGF

There is no correlation between the four indexes in the control group (*P* > 0.05), and netrin-1, DCC and VEGF in the study group are positively correlated but negatively correlated with UNC5B (*P* < 0.05). The correlation of four indicators in the control group is shown in Table 4.

The correlation of four indicators in the research group is shown in Table 5.

### 4.3. Expressions of Netrin-1, DCC, UNC5B, and VEGF Proteins in Villous Tissues

#### 4.3.1. Differences in Positive Expression Rates of the Four Indicators

The positive expression rates of Netrin-1, DCC, UNC5B, and VEGF in villous tissues are shown in Table 6. The positive expression rate of DCC in the study group is lower than that in the control group and the high expression rate of Netrin-1, DCC, and VEGF is lower than that in the control group. The positive expression rate and high expression rate of UNC5B in the study group are significantly higher than that in the control group, with statistically significant differences (*P* < 0.05).

#### 4.3.2. Differences in Relative Expression Levels of the Four Indicators

The protein expression of Netrin-1, DCC, and VEGF in the study group is lower than that in the control group and the protein expression of UNC5B is higher than that in the control group, with a statistical significance (*P* < 0.05). The differences in relative protein expression levels of Netrin-1, DCC, UNC5B, and VEGF are shown in Table 7.

Figure 1 shows the expression of netrin-1 in villous tissues (immunohistochemical staining×400).

Figure 2 shows the expression of DCC in villi (immunohistochemical staining × 400).

Figure 3 shows the expression of UNC5B in villi (immunohistochemical staining × 400).

Figure 4 shows the expression of VEGF in villi (immunohistochemical staining × 400).

### 4.4. Correlation Analysis of Netrin-1, DCC, UNC5B, and VEGF

There is no correlation between the expressions of Netrin-1, DCC, UNC5B, and VEGF in the control group, and the *P* value is higher than 0.05. There is a significant negative association between Netrin-1 and DCC expression in the study group (*r* = −0.332, *P* < 0.001). The expression of DCC and UNC5B is positively correlated (*r* = 0.353, *P* < 0.001). There is no correlation between netrin-1 and UNC5B expression (*r* = −0.034, *P* > 0.05). There is no correlation between VEGF and the expressions of netrin-1, DCC, and UNC5B (*P* > 0.05).

Netrin-1, DCC, and VEGF belong to the positive adjustment factor, which can make the change of placental vascular endothelial cells, migration, and maintain normal pregnancy, and its low expression may result in placental vascular endothelial cell proliferation and migration. The placental villus blood vessels cannot be fully developed, which causes placental vascular area smaller. The blood circulation of the placenta is impaired, and the maternal, fetal nutrition and gas exchange cannot function well, which may lead to delayed abortion. UNC5B is a negative regulator, and the high expression of UNC5B can lead to inhibition of vascular proliferation, migration, and invasion, and disturbance of placental vascular circulation may lead to delayed abortion. These four factors all play a role in the formation and development of placental blood vessels and the remodeling of placental blood vessels, and maintain stable placental blood vessel circulation.

In this study, there are also some shortcomings. Only the protein and mRNA expressions of netrin-1, DCC, UNC5B, and VEGF are detected in the villous tissues of delayed abortion. In the next step, it is necessary to investigate the expression of the above factors in the serum of patients with delayed abortion. If similar trends exist in the serum, whether factors can be prospectively added according to the expression level of each factor in the serum, so as to prevent or relieve placental circulation disorders. It is still necessary to carry out systematic research to verify the above hypothesis.

## 5. Conclusion

In order to investigate the correlation between netrin-1, DCC, UNC5B, and VEGF expression machine in villus tissues of delayed abortion in colorectal cancer, a total of 120 pregnant women were selected from February 2020 to August 2020. The expressions of netrin-1, DCC, VEGF protein, and mRNA in villous tissues of delayed abortion are lower than those of normal pregnant women and the expressions of UNC5B protein, and mRNA is higher than those of normal pregnant women. Such abnormal expressions may be related to the formation disorder of villous blood vessels in the delayed abortion.

## Figures and Tables

**Figure 1:** Expression of netrin-1 in villous tissues (immunohistochemical staining × 400). (a) Control group. (b) Study group.

**Figure 2:** Expression of DCC in villi (immunohistochemical staining × 400). (a) Control group. (b) Study group.

**Figure 3:** Expression of UNC5B in villi (immunohistochemical staining × 400). (a) Control group. (b) Study group.

**Figure 4:** Expression of VEGF in villi (immunohistochemical staining × 400). (a) Control group. (b) Study group.

**Table 1:** Baseline data comparison $\left(\bar{x}\pm s\right)$.

Group	Example number (no)	Age (years)	Pregnancy week (week)	Pregnant times (time)	Number of deliveries (time)
Research group	60	29.15 ± 6.15	10.05 ± 2.11	1.03 ± 0.33	0.98 ± 0.26
Control group	60	30.26 ± 7.11	10.26 ± 2.19	1.12 ± 0.31	1.02 ± 0.24
*t*	—	0.647	0.378	1.089	0.619
*P*	—	0.520	0.707	0.281	0.538

**Table 2:** Primers of the target gene and reference gene.

Primer name	Base sequence (5′-3′)	Product length
*GAPDH*		259
head waters	CATCATCCCTGCCTCTACTGG	
lower reaches	GTGGGTGTCGCTGTTGAAGTC	

*Netrin-1*		197
head waters	ACTGCCATTACTGCAAGGAGG	
lower reaches	GCTCTGCTGGTAGCCTTTGG	

*DCC*		146
head waters	AGCCGATTTGTCCGTCTCAG	
lower reaches	CCCACAGTGAGCTGAAGGGA	

*UNC5B*		194
head waters	GGTCTACTGCCTGGAGGACAC	
lower reaches	GGATCTCCTGGTATTTGGC	

*VEGF*		155
head waters	GAACTTTCTGCTGTCTTGGGTG	
lower reaches	GGCAGTAGCTGCGCTGATAG	

**Table 3:** The PCR results of the four indexes.

Group	Example number	Netrin-1 mRNA	DCC mRNA	UNC5B mRNA	VEGF mRNA
Research group	60	0.64 ± 0.18	0.76 ± 0.22	3.51 ± 0.87	0.95 ± 0.21
Control group	60	1.35 ± 0.31	1.29 ± 0.32	1.34 ± 0.29	2.44 ± 0.38
*t*	—	10.848	7.475	12.961	18.797
*P*	—	<0.001	<0.001	<0.001	<0.001

**Table 4:** Correlation of four indicators in the control group.

Index(r/P)	Netrin-1	DCC	UNC5B	VEGF
Netrin-1	—	0.112/0.326	0.128/0.305	0.201/0.104
DCC	0.112/0.326	—	−0.133/0.244	0.084/0.472
UNC5B	0.128/0.305	−0.133/0.244	—	−0.221/0.087
VEGF	0.201/0.104	0.084/0.472	−0.221/0.087	—

**Table 5:** Correlation of the four indicators in the research group.

index (r/P)	Netrin-1	DCC	UNC5B	VEGF
Netrin-1	—	0.254/0.031	−0.302/0.011	−0.288/0.025
DCC	0.254/0.031	—	−0.288/0.025	0.312/0.009
UNC5B	−0.302/0.011	−0.288/0.025	—	−0.251/0.032
VEGF	0.338/0.003	0.312/0.009	−0.251/0.032	—

**Table 6:** Positive expression rates of Netrin-1, DCC, UNC5B, and VEGF in villous tissues (*n*, %).

Group	Example number	Netrin-1 positive	Netrin-1 high expression rate	DCC positive	DCC high expression rate	UNC5B positive	UNC5B high expression rate	VEGF positive	VEGF high expression rate
Research group	60	24(80.00)	9 (30.00)	10 (33.33)	2 (6.67)	28 (93.33)	25 (83.33)	24 (80.00)	8 (26.67)
Control group	60	27(90.00)	24 (80.00)	28 (93.33)	26 (86.67)	18 (60.00)	5 (16.67)	16 (86.67)	22 (73.33)
*t*		0.523	15.152	23.254	40.431	9.317	26.667	0.480	13.067
*P*		0.470	<0.001	<0.001	<0.001	0.002	<0.001	0.120	<0.001

**Table 7:** Differences in relative protein expression levels of Netrin-1, DCC, UNC5B, and VEGF $\left(\bar{x}\pm s\right)$.

Group	Example number	Netrin-1 protein	DCC protein	UNC5B protein	VEGF protein
Research group	60	0.78 ± 0.22	0.52 ± 0.15	1.82 ± 0.34	0.81 ± 0.23
Control group	60	1.24 ± 0.29	1.09 ± 0.25	1.04 ± 0.21	1.42 ± 0.35
*t*		6.922	1.672	10.691	7.978
*P*		<0.001	<0.001	<0.001	<0.001

## Data Availability

The simulation experiment data used to support the findings of this study are available from the corresponding author upon request.
